The article "Association between Mesenchymal Stem Cells and COVID-19 Therapy: Systematic Review and Current Trends" was published in 2022. Journal: Biomed Res Int.

# Association between Mesenchymal Stem Cells and COVID-19 Therapy: Systematic Review and Current Trends

**DOI:** 10.1155/2022/9346939

**Published:** 2022-06-22

**Authors:** Amaan Javed, Saurab Karki, Zeba Sami, Zuha Khan, Anagha Shree, Biki Kumar Sah, Shankhaneel Ghosh, Sara Saxena

**Affiliations:** ^1^University College of Medical Sciences (University of Delhi), Dilshad Garden, Delhi, India; ^2^Nepalese Army Institute of Health Science, College of Medicine, Kathmandu, Nepal; ^3^Shree Guru Gobind Singh Tricentenary Medical College and Research Institute, Gurugram, Haryana, India; ^4^Public Health Consultant, Uttar Pradesh, India; ^5^B.P. Koirala Institute of Health Sciences, Dharan, Nepal; ^6^Institute of Medical Sciences and SUM Hospital, Bhubaneswar, India; ^7^Dr. D. Y. Patil Medical College, Hospital and Research Centre, Pimpri-Chinchwad, Maharashtra, India

## Abstract

**Background:**

The novel coronavirus first emerged in Wuhan, China, and quickly spread across the globe, spanning various countries and resulting in a worldwide pandemic by the end of December 2019. Given the current advances in treatments available for COVID-19, mesenchymal stem cell (MSC) therapy seems to be a prospective option for management of ARDS observed in COVID-19 patients. This present study is aimed at exploring the therapeutic potential and safety of using MSC obtained by isolation from health cord tissues in the treatment of patients with COVID-19.

**Methods:**

A systematic search was done based on the guidelines of the PRISMA 2020 statement. A literature search was executed using controlled vocabulary and indexing of trials to evaluate all the relevant studies involving the use of medical subject headings (MeSH) in electronic databases like PubMed, Embase, Scopus, *Cochrane Central* Register of Controlled Trials (CENTRAL), and clinicaltrials.gov up to 31 December 2021. The protocol was registered in the PROSPERO register with ID CRD42022301666. *Findings*. After screening finally, 22 remaining articles were included in this systematic review. The studies revealed that MSC exosomes are found to be superior to MSC alone in terms of safety owing to being smaller with a lesser immunological response which leads to free movement in blood capillaries without clumping and also cannot further divide, thus reducing the oncogenic potential of MSC-derived exosomes as compared to MSC only. The studies demonstrated that the lungs healed with the use of exosomes compared to how they presented initially at the hospital. MSCs are found to increase the angiogenesis process and alveolar reepithelization, reducing markers like TNF alpha, TGF beta, and COL I and III, reducing the growth of myofibroblasts and increasing survivability of endothelium leading to attenuated pulmonary fibrosis and even reversing them. *Interpretation*. We can conclude that the use of mesenchymal stem cells or their derived exosomes is safe and well-tolerated in patients with COVID-19. It improves different parameters of oxygenation and helps in the healing of the lungs. The viral load along with different inflammatory cells and biomarkers of inflammation tend to decrease. Chest X-ray, CT scan, and different radiological tools are used to show improvement and reduced ongoing destructive processes.

The article "Association between Mesenchymal Stem Cells and COVID-19 Therapy: Systematic Review and Current Trends" was published in 2022. Journal: Biomed Res Int.

## 1. Introduction

The novel coronavirus first emerged in Wuhan, China, and quickly spread across the globe, spanning various countries and resulting in a worldwide pandemic by the end of December 2019. It followed a course of catastrophic global effects and resulted in more than 3.8 million deaths [1]. This highly contagious viral illness is caused by severe acute respiratory syndrome coronavirus 2 (SARS-CoV-2). The morphology of SARS- CoV-2 consists of a nucleocapsid with helical symmetry surrounded by an envelope. The single-stranded viral RNA genome is responsible for causing enteric and respiratory diseases in humans and is mainly transmitted via respiratory droplets, aerosols, and contact routes. The virus enters the body by binding its spike glycoprotein antigen with the host cell receptor called angiotensin-converting enzyme 2 and thus gains entry inside host cells via endocytosis [2]. Typically, the patient can present with common symptoms such as fever, nonproductive cough, dyspnoea, fatigue, myalgia, rhinorrhea, sore throat, and diarrhoea. The patients experiencing dyspnoea usually require intensive care as the body elicits an immune response to fight off the virus through antigen-presenting cells; they are presented to CD8 T cells and natural killer cells by incorporating into the major histocompatibility complex. Thus, both the innate and adaptive immune systems of defence are activated, releasing large numbers of cytokines which may manifest as cytokine storm in certain patients. Cytokine storm is largely responsible for the series of diverse local and remote signs associated with the infection. As the disease progresses acute respiratory distress syndrome (ARDS), acute cardiac injury, secondary infection resulting in generalized sepsis, and multisystem failure might ultimately result in high mortality rates [3]. Given the current advances in treatments available for COVID-19, mesenchymal stem cell (MSC) therapy seems to be a prospective option for the management of ARDS observed in COVID-19 patients. The cells exert potent modulatory effects on lungs and other tissue as they work by reducing and healing inflammation-induced injuries. Since ARDS is known to be one of the leading reasons for death in COVID-19 patients accompanied by hallmarks of cytokine storm, suppression of its aggravation might diminish the provocative cytokine production and subsequently decrease inflammation and lung injury. The immunological trademark comprises lymphopenia and a flurry of active molecules, largely dominated by interleukin IL-6 and tumour necrosis factor TNF-*α* [4]. As per a new declaration of the International Society for Stem Cell Research (ISSCR), at present, there are no endorsed stem cell-based methodologies for the counteraction of coronavirus disease. In any case, as of late, mesenchymal stem cells (MSCs) have presented one of the restorative methodologies for utilizing in the treatment of COVID-19 [5]. MSCs in general were first used as cellular therapy back in 1995 and have since been used in basic research and clinical applications [6] in cases of autoimmune disease, graft-versus-host disease (GVHD), and other diseases with very good safety rates. They assume a positive part in immunomodulatory effects through releasing many types of cytokines by paracrine secretion or making direct collaborations with immune cells. Among these, the human umbilical cord Wharton's jelly-derived MSCs (hWJCs) can be easily obtained and cultured. Inferable from their strong immunomodulatory capacity, hWJC transplantation might forestall or lessen the cytokine storm [4]. Thus, out of all the potential treatments, mesenchymal stem cell (MSC) therapy seems to be a promising option for the management of ARDS seen in COVID-19 patients. Therefore, this present study is aimed at exploring the therapeutic potential and safety of using MSC obtained by isolation from health cord tissues in the treatment of patients with COVID-19.

The article "Association between Mesenchymal Stem Cells and COVID-19 Therapy: Systematic Review and Current Trends" was published in 2022. Journal: Biomed Res Int.

## 2. Methods

### 2.1. Study Strategy

In this study, a systematic search was done based on the guidelines of the Preferred Reporting Items for Systematic Reviews and Meta-Analyses (PRISMA 2020 statement) [7]. The data was collected and organised concerning synthesis without meta-analysis (SWiM) guidelines. A literature search was executed using controlled vocabulary and indexing of trials to evaluate all the relevant studies involving the use of medical subject headings (MeSH) in electronic databases like PubMed, Embase, Scopus, *Cochrane Central* Register of Controlled Trials (CENTRAL), and clinicaltrials.gov up to 31 December 2021. The protocol was registered in the PROSPERO register with ID CRD42022301666. The literature search was carried out using the following search keyword strategy:

*MEDLINE*: (COVID.mp. OR COVID-19.mp. OR coronavirus disease 2019.mp. OR 2019-nCoV.mp. OR severe acute respiratory syndrome coronavirus 2.mp. OR SARS-CoV-2.mp.) AND (mesenchymal stem cells.mp. OR exp mesenchymal stem cells/] OR [exp MSC/OR MSC.mp.] OR [stem cell.mp. OR exp stem cell/] OR [exosomes.mp. OR exp exosomes/]

*EMBASE:* (COVID OR COVID 19 OR coronavirus disease 2019.mp. OR 2019-nCoV.mp. OR SARS-CoV-2.mp. OR severe acute respiratory syndrome coronavirus 2.mp.) AND (mesenchymal stem cells.mp. OR exp mesenchymal stem cells/] OR [exp MSC/OR MSC.mp.] OR [stem cell.mp. OR exp stem cell/] OR [exosomes.mp. OR exp exosomes/]

*Scopus:* (TITLE-ABS-KEY (COVID OR COVID 19 OR [coronavirus AND disease 2019] OR 2019-nCoV OR SARS-CoV-2 OR [severe AND acute AND respiratory AND syndrome AND coronavirus 2]) AND TITLE-ABS-KEY (mesenchymal stem cells OR stem cells OR [cells AND exosomes]

*Cochrane Central:* COVID AND (neuro∗ OR brain OR peripheral nerve OR cerebrospinal fluid)

*Clinicaltrials.gov:* Recruiting and not yet recruiting trials involving the use of mesenchymal stem cells in the treatment of COVID-19

### 2.2. Study Selection

The inclusion criteria considered in this systematic review were full-text articles with (a) English language, (b) the preceding search strategy, (c) requisite information, and (d) reported outcomes on the therapeutic efficacy of mesenchymal stem cells on COVID-19. The exclusion criteria were (a) duplicates, (b) poster, (c) not related to paper, (d) editorials, and (e) letter to the editor.

### 2.3. Data Extraction

Each eligible article will be reviewed, and the following data are extracted: (a) author name and relevant details; (b) outcomes of MSC stem cells and their derived exosomes on COVID-19; (c) study type; and (d) reported symptoms. The clinical trials included were analyzed for: identifier, study title, phase, subjects, cell therapy, route of administration, intervention, and efficacy.

## 3. Result

### 3.1. Literature Review

The process of study selection is illustrated in Figure 1.

909 articles were obtained by searching the aforementioned databases using the mentioned search keyword strategy. After the screening articles, 842 of them were excluded using the exclusion criteria by evaluation and abstracts, and 48 studies were qualified for assessment of their full-text. Thereafter, the studies still inconsistent with inclusion criteria were omitted. Finally, 22 remaining articles were included in this systematic review: Table 1 contains summary data extracted from these studies with the use of MSC therapy in cases of SARS-CoV-2 infection.

### 3.2. Therapeutic Efficacy of MSC and MSC Exosomes

MSC therapy has given hope for treating various autoimmune disease conditions. MSCs are nonhematopoietic cells that have immune-modulatory, regenerative, and differentiation properties [8, 9]. MSCs were first tested as cellular therapy in humans in 1995 and have since been used in basic research and clinical applications [10]. Due to the immunomodulatory properties possessed by mesenchymal stem cells, there has been growing evidence of its utility in offering a possible line of treatment for various diseases for which no reliable and efficacious treatment exists to date. The diseases for which MSC therapy holds a ray of hope are majorly autoimmune disorders. Hafsa Munir and Helen M McGettrick reviewed the clinical trials done on the effect of MSC therapy on Crohn's disease, systemic lupus erythematous, and rheumatoid arthritis and revealed potent immunomodulatory effects in all the trials [11]. Although no adverse effects were reported, the mechanism of action of MSC needs more clarity. Chen et al. tested the effects of different treatments in a mouse model of experimental autoimmune hepatitis (EAH) and found that administration of culture-expanded bone marrow-derived MSCs can reduce EAH in a dose-dependent way, and the therapeutic effect observed in the group that received an intravenous (IV) injection three times was better than a single injection [12], whereas Wang et al. reported that both IL-35 gene-modified MSCs (IL-35-MSCs) and adipose-derived MSCs have a protecting effect in induced fulminant hepatitis in mice models. They reported that IL-35-MSCs exerted a therapeutic impact more powerful than adipose-derived MSCs [13]. Several experimental studies provide evidence that MSC derived from bone marrow has the potential for being effective in treating critically ill surgical patients who develop traumatic brain injury, acute renal failure, or acute respiratory distress syndrome. There is also preclinical evidence that MSC may be effective in treating sepsis-induced organ failure, including evidence that MSC has antimicrobial properties [14]. In humans, the most studied application for MSCs is graft—versus—host disease (GVHD). GVHD is a condition in which a genetically dissimilar, immunocompromised recipient gets attacked by the donor T cells after getting a hematopoietic stem cell transplantation [15]. Another clinical trial involving Crohn's disease (CD) resulted in the healing of fistulas with no adverse effects when treated with MSC injections [16, 17]. Perhaps the most remarkable results of human MSC therapy emerge now from clinical trials aimed at severe, treatment-refractory systemic lupus erythematosus (SLE) [18–21]. Thus, the number of preclinical and clinical studies on patients and various experimental studies done on animal models support MSC therapy as the way forward. The properties of MSC are illustrated in Figure 2.

The article "Association between Mesenchymal Stem Cells and COVID-19 Therapy: Systematic Review and Current Trends" was published in 2022. Journal: Biomed Res Int.

### 3.3. Immunomodulation Mechanism of MSCs

Mesenchymal stem cells can divide into various cell types, like *β* cells of islets of Langerhans in the pancreas, cardiac myocytes, fat cells, osteoblasts, and, conceivably, nerve cells. Apart from their differentiation ability, MSCs have been known to monitor the immune response in several conditions. It has been reported that adult MSCs can modify the T cell and B cell responses [22]. They improve tissue repair and regeneration by changing the immune response, and they work as modulators of inflammation instead of renewing the injured cells [23]. Immunomodulatory effects of both innate and adaptive immunity can be generated by MSCs. They suppress T cell production and cytokine release, including mediators such as IL-10, TGF *β*, indoleamine 2,3-dioxygenase, and PGE2, and they also limit the differentiation of dendritic cells, increasing the quantity of Tregs and suppressing the effector T cells via multiple growth factors, iNOS, heme oxygenase-1, prostaglandin E2 (PGE2), and indolamine-2,3-dioxygenase (IDO) [24]. Cytokine storm leads to a rigorous inflammatory reaction due to the body's overactive immune system, which initiates focally and then spreads to the systemic circulation, causing damage to various organs in the body. Apart from COVID-19 infection, cytokine storm is also observed in infectious diseases due to SARS-CoV, influenza, Epstein-Barr virus, variola virus, and streptococci. It was originally seen in the graft-vs.-host disease during organ transplants [25]. MSCs can move to the damaged tissue. In the injured lung, acute respiratory distress syndrome, and sepsis, MSCs travel to and are confined in the lungs, leading to the release of growth factors, antimicrobial factors, and cytokines [26]. It even causes the reduction of apoptosis of various cells by the expression of TNF-alpha, IL-1, and IL-6 [27]. Disease caused by Th2-driven immune response has been decreased by the use of multipotent adipose-derived stem cells, a type of MSCs. It produces immunosuppressive effects by modulating both cellular and immune pathways. It inhibits Th2-dependent airway allergic diseases [28]. MSCs derived from bone marrow are found to inhibit Th2-mediated airway inflammation by causing CD4 cell differentiation which decreases lung inflammation mediated by Th2 through IFN-gamma dependent process [29]. In one of the study, gingivae-derived MSCs was able to reduce both clinical and histopathological severity of colonic inflammation and was able to reduce the inflammatory infiltration of T cells and expression of anti-inflammatory cytokine like IL-10 [30]. Suppression of antigen-specific cell Th1/Th17 decreases the production of inflammatory cytokines, and production of CD4+, CD25+, FoxP3+, and regulatory T cells suppresses self-reactive T cells which has been possible from the adipose-derived MSCs because it has been used in inflammatory conditions [31]. MSC activity has not only been limited to regeneration but the immunomodulatory and inflammatory property has heightened its importance in modern medicine. The use of MSC stem cells and their derived exosomes concerning other therapeutic roles has been discussed in the subsequent sections.

The article "Association between Mesenchymal Stem Cells and COVID-19 Therapy: Systematic Review and Current Trends" was published in 2022. Journal: Biomed Res Int.

#### 3.3.1. Wound Healing and Soft Tissue Defects

Optimal wound healing involves three overlapping phases: inflammation, proliferation, and resolution. The inflammatory phase is initiated by a microorganism or toxin that leads to the release of pathogen/damage-associated molecular patterns (PAMPs/DAMPs, respectively) that activate Toll-like receptors, NOD-like receptors (NLRs), and C-type lectin receptors (CLRs) on host cells. Interaction of these receptors causes the synthesis and release of GFs, cytokines, and chemokines that cause the migration of inflammatory cells, principally neutrophils, and monocytes. The monocytes reach the tissue and eventually develop into macrophages. Inflammatory macrophages and host cells generate reactive oxygen species that kill microorganisms [32]. Moreover, they promote the gene expression of numerous cytokines, inflammatory cells, and various proteases such as matrix metalloproteinases, serine, cysteine proteases, and elastases. These effects are caused by a variety of mechanisms, including changes in the balance of proinflammatory and anti-inflammatory cytokine release. Proinflammatory transcription factors necessary for neutrophil survival, such as NF-*κ*B and IRF1, are downregulated [33], whereas the anti-inflammatory transcription factor IRF-4 is upregulated, eventually leading to the resolution of the inflammatory phase and initiation of the tissue repair phase. Fibrosis-promoting macrophages appear at this phase, either by the differentiation of newly recruited infiltrating monocytes or through the in situ transformation of previously differentiated infiltrating inflammatory macrophages to a profibrotic type. During this change, there is an activation of STAT6 which promotes IL-4/IL-13-mediated differentiation of profibrotic macrophages by upregulating the expression of arginase and other profibrotic phenotypic genes. Profibrotic macrophages elicit the activation of fibroblasts to increase extracellular matrix synthesis and secretion. The scar tissue is reformed in the last phase by replacing friable type III collagen with durable and long-lasting type I collagen by significant collagen cross-linking. These modifications are followed by the death of active myofibroblasts and decreased neovascularization. Adipose-derived stem cells (ASCs) are found in the stromal vascular fraction (SVF) of subcutaneous fat tissue. It contains a diverse group of mesenchymal cells. These cells can be separated further by using enzymatic digestion to remove most of the hematopoietic cells from the SVF cells or by combining the filtering and centrifugation procedures as mechanical digestion. ASCs-SVFs can enhance the fibrogenic activity of fibroblasts, which promotes vascularization by enhancing fat tissue survival and 3D organization/ASCs express proangiogenic factors like vascular endothelial growth factor (VEGF), interact with blood vessels perivascularly, and offer physical extracellular matrix guiding signals that lead to endothelial growth [33].

The article "Association between Mesenchymal Stem Cells and COVID-19 Therapy: Systematic Review and Current Trends" was published in 2022. Journal: Biomed Res Int.

#### 3.3.2. Hair Regrowth

To ameliorate the problem of alopecia and enhance hair growth, hair bioengineering has risen to the next level demonstrating new approaches for it. The mesenchymal stem cells are the solution to many problems and can be used even in the treatment of these problems too. Human intra and extradermal adipose tissue-derived hair follicle stem cells (HD-AFSCs) contain hair follicle mesenchymal stem cells (HF-MSCs), and hair follicle epithelial stem cells (HF-ESCs) can be used for the advancement of hair growth [34]. HF-MSCs show positive staining for CD44, CD73, CD90, and CD 105 which are the surface markers of bone marrow mesenchymal stem cells which has the potential to differentiate [35]. Gentile showed the HD-AFSCs show positivity for CD44, CD100, CD200, and S100A4 which represent the early progeny of stem cells and help in the expression with the growth of keratinocytes [34]. MSC cells express Wnt/*β*-catenin signalling molecules which have been shown as a fundamental factor that augments hair growth [36, 37]. There also occurs expression of VEGF, TGF-*β*, IGF-1, IGFBP-1to-6, M-CSF, M-CSFR, PDGF, PDGFR-*β*/-*α*64, PGE2, and PGF2 *α* which all contributes in the hair regrowth [38]. Dermal papilla cells (DPCs), a part of autologous stem cells, also play role in the regulation of hair growth and regeneration [38]. DPCs secrete alkaline phosphate which is required in the early anagen period [39]. It expresses *α*-smooth muscle actin and versican which are the marker of the dermal papilla and helps in the induction and maintenance of hair growth [40, 41]. It even expresses CD133 which is a stem cell marker and promotes hair follicle neogenesis. The application of MSCs in hair growth would lead to a breakthrough revolution in alopecia. More clinical trials and research are required in this field.

The article "Association between Mesenchymal Stem Cells and COVID-19 Therapy: Systematic Review and Current Trends" was published in 2022. Journal: Biomed Res Int.

### 3.4. COVID-19 Pathophysiology

COVID-19 is a viral disease caused by SARS-Cov-2 which appeared in Wuhan of China around December 2019 [42]. The virus is an enveloped single-stranded RNA virus that enters the host cell through angiotensinogen converting receptor 2 [43]. The infection can affect the respiratory system, both the upper and lower, ranging from asymptomatic acute infection to subacute and chronic infection leading to fibrosis and scars as well as the dreadful acute respiratory distress syndrome along with multiple organ failure. Besides the respiratory system, it can affect multiple organs and tissues leading to complications like meningitis, encephalitis, myocarditis, acute renal failure, venous thromboembolism, and many more [44]. The virus primarily transmits through saliva, droplets, or respiratory secretions. It enters the cells through the ACE-2 receptor by binding to spike glycoprotein and thus gains entry inside the cells. The host immune system then identifies antigens of the virus, and through antigen-presenting cells, they are presented to CD8 T cells and natural killer cells by incorporating them into a major histocompatibility complex. Thus, both innate and adaptive immune systems of defence are activated. However, in some individuals, the production and secretion of cytokines are massive leading to cytokine storm which leads to coagulopathy and multiple organ failure resulting in death [45]. Another hypothesis that has been explained regarding the pathogenesis of COVID-19 is regrading inhibition of human heme metabolism. The RNA virus has been presumed to bind the beta chain of the porphyrin moiety of red blood cells and thus impairing heme metabolism as well as the release of iron which needs further study to confirm [46]. Multiple cytokines have been associated with COVID-19 infection like TNF alpha, IL-1 beta, and IL-8; however, there has been particular interest in IL 6. The cytokine has been associated with various types of tissue injury like burns, trauma as well as septic shock, and in the case of COVID-19, it has a vital role in the development of cytokine release syndrome [47]. This cytokine which normally plays a role to defend against tissue injuries and infections has also been found to be among the highest level among cytokines associated with severe and critical infection [48]. Thus, tocilizumab, a monoclonal antibody against IL-6, has a therapeutic role that decreases the chance of reducing the combined consequence of mechanical ventilation and demise [49, 50]. TNF alpha is another cytokine that also has been widely studied for its tissue-damaging role in cytokine release syndrome. It is produced by different inflammatory cells like macrophages, T cells, and epithelial cells, and it functions to recruit neutrophils at the site of inflammation-causing airway inflammation and hyperreactivity [51]. Another important context to discuss regarding the pathogenesis of COVID-19 is the role of the exosome. Exosomes, which are membrane vesicles, are released due to the fusion of the organelle following endocytosis with the plasma membrane [52]. It is believed that the protein of SARS CoV 2 protein interacts with the Rab proteins which is a component of the ESCRT (endosomal sorting complex required for transport) pathway which has a role in the synthesis of exosomes [53]. Similarly, with ganglioside (GM3) enrichment of the exosomes, it was found to be related to the disease severity and probable cause for lymphopenia, as the cells of the immune system would prefer exosomes with GM3 enrichment and thus leading to cellular cytotoxicity [54]. Most viruses are believed to enter the exosome during the synthesis of virion particles as well as spread to the naïve host cells which are not seen in SARS CoV 2, though the experimental studies are present to show that the virus exists in two-layered membrane vesicles. It is thus these extracellular vesicles and the exosomes which might be the potential mediators for infection, reinfection, and subsequent reactivation of the viral particles [55]. The first virus strain that appeared in the seafood market of Wuhan of China and the subsequent strains found in Italy differed in terms of mutation in the spike protein, precisely a missense mutation of aspartate for glycine at 614 (D614G) position and thus account for the difference in demographics factor as well as the viral lethal nature [56]. Similarly, the UK variant (201/501Y.Vq) had S: N501 mutation at RDB (receptor binding domain) which might result in higher binding of spike protein to ACE2. South African (20H/501Y.v2) strain and Brazilian (20J/501Y.V3) strain both had mutation S: E484 at the RDB location resulting in a similar role as the British variation [57]. Then, Delta variant with mutation such as E484Q, P614R, and L452R resulting in easier binding of spikes protein to the ACE-2 receptor, which emerged in India and replaced the existing variant of concerns, Alpha variant that was first reported in the UK, Beta variant of South Africa, and Gamma variant of Brazil, was associated with increased disease severity and rate of viral transmission and was also associated with infections among the vaccinated individual [58, 59]. It is thus important to know the viral pathogenesis and different mutations to ensure that a proper vaccination will work and prevent transmission among individuals to reduce the public health issue that the virus has imposed and the global burden of the ongoing pandemic. The process of action of MSC on patients suffering from SARS-CoV-2 is illustrated in Figure 3.

The article "Association between Mesenchymal Stem Cells and COVID-19 Therapy: Systematic Review and Current Trends" was published in 2022. Journal: Biomed Res Int.

### 3.5. COVID-19 concerning MSC and Their Derived Exosomes

MSC cells present with multiple biological properties, which include high regenerative capacities and the ability to augment tissue repair [60], but most importantly the cell's ability to control and modulate immune responses is the reason why they are currently being investigated in several clinical diseases to establish them as cellular therapy tools in cases of inflammatory diseases [61]. These cells do not trigger any host responses that can lead to cell rejection thus making them the safer option of all the other kinds of stem cells available. Mesenchymal stem cells (MSCs) are already being used for the treatment of autoimmune disorders, type 2 diabetes, spinal cord injury, and other diseases [62, 63]. The cells are also the suggested potential treatment for H5N1 infection responsible for inducing acute lung injury, similar to what is observed in COVID-19 with inflammatory cytokines [64]. The presence of SARS-CoV2 in the lung induces an uncontrolled generalized immune response. Various immune cells like neutrophils, T-lymphocytes, and macrophages are recruited to the lungs. The leading cause of mortality in COVID-19 patients is hypoxemic respiratory failure, which results in acute respiratory distress syndrome (ARDS). When administered intravenously, the cells are trapped within the lung's capillary beds in a short duration of action, allowing efficient delivery of MSC cells in the lungs making it beneficial in cases of ARDS involving COVID [65–67]. They mitigate the effect of viral disease due to the presence of specific cytokines. MSCs can decrease cytokine storm, replace injured alveolar epithelial cells, and facilitate tissue repair by secreting anti-inflammatory cytokines and antifibrotic growth factors, suppress and modulate immune responses, lower inflammatory effects, and protect the epithelial lining of alveoli during ILI and acute respiratory distress syndrome [68]. Therefore, the immunomodulatory functions of stem cells and MSC exosomes can potentially enable us to use them as a treatment for COVID-19 [69]. As the pandemic is pacing, it is essential to consider various therapeutic options to treat the population. Since the immune system is the main target of the infection, we need to maintain a balance to prevent the exaggerated immune responses that eventually lead to multiorgan failure. The cells stop pulmonary fibrosis, heal the pulmonary circuit and alveolar epithelial lining, treat lung collapse and SARS-CoV 2 associated pneumonia, and improve the overall lung function [70]. Several clinical trials reported the effectiveness and safety of MSCs sequestered from plenty of allogeneic sources. It was noticed that after one dose of stem cell infusion, there was considerable progress in the conditions of these patients without any damaging effects. After two days of stem cell transplantation, there was marked progress in the respiratory functioning of these subjects [71]. During the clinical trials for the treatment of severely ill patients who had COVID-19-induced ARDS, the majority of the cases who recovered responded substantially in about 48 to 96 hours after the initial infusion of stem cells. The patients who survived were in good health throughout the follow-up evaluation for 60 days. The only adverse effect was temporary shivering and chills, which happened initially in two patients. The shivering was not linked with fever and COVID-19 infection, and it ceased in an hour with the help of supportive treatment [60]. Upon further investigation, the lab findings showed an elevated inflammatory response accompanied by severe thrombocytopenia, D-dimer levels were also found to be high. There were no known signs of pulmonary embolism in the CT pulmonary angiography but there was a progression of bilateral consolidations [72]. Overall, no improvement was observed in radiological findings, CT scan images, and histological findings after the administration of umbilical-cord blood-mesenchymal stem cells (UCB-MSCs), but there was significant consolidation of the lungs which progressed into diffuse lung fibrosis, which commonly occurs in critical COVID-19 patients. Pulmonary fibrosis comes under the category of increasing interstitial pneumonia that occurs due to an exaggerated response of chronic inflammation and healing wound. It is usually started by recurrent injury to the epithelium [73]. MSC cells use and safety profile also requires monitoring in patients with COVID-19 while undergoing treatment because of the multisystem nature of the disease associated with coagulopathy [74]. Another study conducted in Hubei Province where patients were divided into two groups found that of the 12 patients who were treated with hUC-MSC, there was no need for invasive ventilation. No patient progressed from severe to critical illness as the 28-day mortality rate was found to be zero but in the control group, the results were the opposite, in a total of four patients. They progressed to critical illness and, as a result, had to receive invasive ventilation out of which three patients died; hence, the 28-day mortality was calculated to be 10.34%. Although in comparison the differences were not very significant, the improvement trend could be easily traced. In light of this information, it is safe to believe that if the sample size is large, there could be significant differences [75]. Moreover, a noninvasive treatment, hUC-MSC therapy, is a very effective and promising method for clinical application.  Table 2 contains a summary of clinical trials recruiting and not yet recruiting aiming to use MSC and their derived exosomes for COVID-19 therapy.

The article "Association between Mesenchymal Stem Cells and COVID-19 Therapy: Systematic Review and Current Trends" was published in 2022. Journal: Biomed Res Int.

### 3.6. Biomolecular Basis of AD-MSCs and Application in COVID-19

Adipose-derived stem cells (ASCs) are a type of mesenchymal stem cells (MSCs) that can be easily obtained from adipose tissues. They possess regenerative properties similar to that of other MSCs. ASCs differentiate into multiple cell lineages, offering the potential to repair, maintain, or enhance various tissues. They contain various types of cells like preadipocytes, adipocytes, macrophages, endothelial cells, and smooth muscle cells supported by connective tissue and fine capillaries. ASCs have been shown to demonstrate the ability to proliferate in a culture medium greater than other MSCs. Various receptor pathways regulate ASC proliferation and differentiation. FGFRs and the ErbB tyrosine kinase receptor family are involved in the control of both the growth and differentiation of ASCs [76, 77]. Increased Akt activity plays a crucial role in this process, as well as through the parallel downregulation of EGFR and ErbB2 expression, and Erk-1 activity [78]. Also, it is known that the degree of tissue growth and regeneration is based on the level of formation of new blood vessels known as neoangiogenesis [79]. Studies suggest that neovascularization and adipogenesis interact through paracrine signalling and occur in a coupled manner throughout adult life. Recent studies indicate that ASCs and MSCs are capable to promote neoangiogenesis through the secretion of growth factors, in particular VEGF [79–81]. Since human adipose tissue is easily obtained in large quantities using a minimally invasive procedure, the use of autologous ASCs is promising for both regenerative medicine and organs damaged by injury and disease, leading to a rapidly increasing field of research.

The application of stem cells as potential therapeutic strategies has shown promising results in vitro experiments and preclinical studies. After bone marrow, adipose tissue is regarded as the most estimable source for the cultivation of MSCs, with a total estimate of 98–100% cell viability [82]. The large quantity and facile access to the cells via liposuction procedures prove to be of great advantage when combating COVID-19-induced pneumonia. Thirteen such severe cases of COVID-19 consisting of patients under invasive mechanical ventilation support were administered doses of allogenic adipose stem cells. These cases later presented favourable clinical and biological outcomes. Another study conducted by Zheng et al. to demonstrate the safety of intravenous administration of allogeneic ASCs in patients with ARDS resulted in a short-term improvement of oxygenation in the body [83]. In most clinical cases, no adverse events were reported concerning cell therapy. The treatment with AT-MSC showed a decrease in levels of inflammatory parameters (C-reactive protein, IL-6, ferritin, LDH, and d-dimer) along with an increase in lymphocytes, especially in the patients who showed clinical improvement [84]. These results comply with ASCs' ability to differentiate into multiple cell lineages along with the secretion of various cytokines, and other immunomodulatory properties [85]. These adipose tissue grafts typically involve a minimum of two cell type mature adipocytes and stromal vascular fraction (SVF). SVF incorporates endothelial cells, smooth muscle cells, leukocytes, mast cells, preadipocytes, pericytes, and multipotent adipose-derived stem cells (ASCs) coming together to form a heterogeneous cell population [86]. Other studies have highlighted the potential use of AD-MSCs in regeneration of damaged tissue through the use of exosomes and microRNAs. The excessive secretory action by SVFs and AD-MSCs makes them a fitting vehicle for the delivery of drug molecules in the cellular microenvironment [87]. The results of antimicrobial activity of mesenchymal stem cells carried out by Francisca A. Miranda provides credible insights into adipocyte-secreted exosomal microRNA (A-SE-miR) function and potential use as an antiviral [88]. On this basis, ASC treatments may reduce the demand for critical hospital resources in COVID-19 patients.

The article "Association between Mesenchymal Stem Cells and COVID-19 Therapy: Systematic Review and Current Trends" was published in 2022. Journal: Biomed Res Int.

## 4. Discussion

From our studies which include 22 analyzed studies with the use of mesenchymal cells and their derived exosomes and 17 ongoing clinical trials involving the use of mesenchymal cells in the treatment of COVID-19, significant data involving therapeutic use of MSCs concerning COVID-19 was extracted. Out of those analyzed studies, four studies demonstrated that the use of mesenchymal cells and their exosomes are found to be safe and well-tolerated by patients with COVID-19. It is to be noted that MSC exosomes are found to be superior to MSC alone in terms of safety owing to being smaller with a lesser immunological response which leads to free movement in blood capillaries without clumping and also cannot further divide, thus reducing the oncogenic potential of MSC derived exosomes as compared to MSC only [89]. Improvement in oxygenation was shown in four studies. These oxygenation parameters are reported in terms of improved SpO2 following infusion of MSC, decreasing FiO2 with improved PaO2 and SaO2, PaO2/FiO2 ratio, and oxygenation index. Six studies demonstrated that the lungs healed with the use of exosomes compared to how they presented initially at the hospital. MSCs are found to increase the angiogenesis process and alveolar reepithelization, reducing markers like TNF alpha, TGF beta, and COL I and III, reducing the growth of myofibroblasts and increasing survivability of endothelium leading to attenuated pulmonary fibrosis and even reversing them [90]. Similarly, two studies focused on the improvement of renal function. As many as eleven studies showed that there was a significant reduction in inflammatory cells and inflammatory markers. A review by Shetty et al. demonstrated that the use of mesenchymal cells can increase the release of different factors leading to protection of epithelium of alveoli with decreased fibrosis and hence better lung physiology [60]. Such cells are responsible for decreasing inflammatory response, with regulated immunity ultimately leading to protection of respiratory cells at times of severity like ARDS and acute lung injury [71]. Improvement of radiological presentation as clearing of CT findings of bilateral lung exudate or ground-glass opacity or chest X-ray findings was demonstrated by six studies. Two studies demonstrated that the use of exosomes could reduce the deadly cytokine storm. With the combined efforts of the proliferation of the epithelium, modulated immune response, and removal of excess fluid from alveoli, this can reduce the damage induced by the virus in lung parenchyma as well as the body systems leading to a reduction in the cytokine storm. As many as 12 studies demonstrated that mesenchymal stem cells do have an important role to improve patients' survival and reduction of mortality. As for ongoing registered clinical trials, four of them will be focusing on oxygen saturation following the use of exosomes. Six of the clinical trials will look for treatment-emergent adverse effects during therapy.

## 5. Conclusion and Future Perspectives

From this review, we can conclude that the use of mesenchymal stem cells or their exosomes is safe and well-tolerated in patients with COVID-19. It improves different parameters of oxygenation and helps in the healing of the lungs. The viral load along with different inflammatory cells and biomarkers of inflammation tends to decrease. Chest X-ray, CT scan, and different radiological tools are used to show improvement and reduced ongoing destructive processes. Similarly, the severe form of COVID-19 infection, ARDS, and different complications of a cytokine storm are attenuated following MSC therapy. Thus, it tends to reduce morbidity and mortality leading to improved inpatient survival and reducing the length of ICU stay. MSC and MSC like derivatives are found to have shown promising results in terms of safety and suitability in the early stage of initiation. Exosomes that are released from MSCs are currently a novel way to treat COVID-19 infection owing to their role in immune system modulation and regenerative characteristics. Our systemic review has several limitations like there is only a small number of studies that have been recruited in the review. Each study has its heterogeneity in the design of studies and demographics of the population included. Similarly, each included studies have its limitations. Further, cohorts and randomised controlled trials with a larger sample size in this particular field of interest should be done to uncover the reality of its effect in COVID-19. Larger cohorts and clinical trials with greater sample sizes are required to uncover the current findings like its efficacy, potency, and timing of dosing with even greater consistency and accuracy. Similarly, additional emphasis should be given to standardizing the treatment and building protocols to upgrade the standard of care in the ongoing pandemic. Ongoing clinical trials should be completed properly to add something to the existing literature as well as in patient care.

The article "Association between Mesenchymal Stem Cells and COVID-19 Therapy: Systematic Review and Current Trends" was published in 2022. Journal: Biomed Res Int.

## Figures and Tables

**Figure 1:** Process of study selection based on Preferred Reporting Items for Systematic Reviews and Meta-Analyses (PRISMA 2020 statement).

**Figure 2:** Summary of properties of MSC exosomes.

**Figure 3:** Summary of actions of MSC and their derived exosomes on patients with COVID-19.

**Table 1:** Summary of studies analysed for use of MSC and their derived exosomes for SARS-CoV-2 infection.

Reference	Therapy used	Intervention	Outcome
Ciccocioppo et al. [91] (*n* = 1)	Cell therapy	1.1 × 10^6^ cells/per kg body weight of MSCs	Improvement of the inflammatory, respiratory, thrombotic, and renal parameters was observed after 2 and 8 days after MSC infusion
Senegaglia et al. [92] (*n* = 1)	Tocilizumab and allogenic umbilical cord-derived mesenchymal stromal cells	Infusion of 400 mg of tocilizumab and three intravenous infusions of 500,000 Cells per kilogram in alternate days	The relative viral quantification decreased gradually from day zero and was undetectable in day 14
Shu et al. [75] (*n* = 41)	Standard treatment plus umbilical cord mesenchymal stem cell infusion vs. standard treatment	2 × 10^6^ cells/kg of MSCs suspended in 100 mL of normal saline	CRP and IL-6 levels were significantly lower from day 3 of infusion, the time for the lymphocyte count to return to the normal range was significantly faster, and lung inflammation absorption was significantly shorter on CT imaging in the hUC-MSC group than in the control group.
Xu et al. [93] (*n* = 44)	MSC transplantation along with comprehensive treatment vs. comprehensive treatment only	Three infusions totaling 9 × 10^7^ MSCs every other day (day 1, day 3, and day 5). Each infusion contained 3 × 10^7^ cells resuspended in 500 mL saline solution	There was a significant improvement in dyspnea while undergoing MSC infusion on days 1, 3, and 5. Additionally, SpO2 was significantly improved following MSC infusion, and chest imaging results were improved in the experimental group in the first month after MSC infusion.
Feng et al. [94] (*n* = 28)	Human umbilical cord mesenchymal stromal cells along with standard treatment vs. standard treatment	2 × 10^6^ cells/kg of MSCs suspended in 100 mL of normal saline	Intravenous transplantation of hUC-MSCs accelerated partial pulmonary function recovery and improved HRQL, indicating relative safety and preliminary efficacy of this treatment for patients with severe COVID-19
Shi et al. [95] (*n* = 100)	UC-MSC vs. placebo	UC-MSC at dose 4∗10^7^ cells per infusion on day, 0, 3 and 6 vs. placebo	UC-MSC administration was safe and well tolerated and exerted a trend of improvement in whole lung lesion and significantly increased the resolution of lung solid component lesions compared with the placebo.
Sengupta et al. [96] (*n* = 27)	Exosomes (ExoFlo) derived from allogeneic bone marrow mesenchymal stem cells	15 mL of ExoFlo was added to 100 mL of normal saline	Laboratory values revealed mean reduction by 32% in neutrophil count, average CD3+, CD4+, and CD8+ lymphocyte counts increasing by 46%, 45%, and 46%, respectively. Likewise, acute phase reactants declined, with mean C-reactive protein, ferritin, and D-dimer reduction of 77%, 43%, and 42%, respectively.
Liang et al. [97] (*n* = 1)	Human umbilical cord mesenchymal stem cells	Allogenic hUCMSCs given 3 times (5∗10^7^ cells each time) with a 3-day interval at days 13, 16, and 19, together with thymosin a1 and antibiotics daily injection	After these treatments, most of the laboratory indexes and CT images showed remission of the inflammation symptoms. The counts of CD3+ T cell, CD4+ T cell, and CD8+ T cell remarkably increased to the normal level, indicating the reversal of lymphopenia.
Haberle et al. [98] (*n* = 23)	Mesenchymal stromal cells	One million MSCs/kg body weight was infused over 30 minutes, and the process was repeated in 3 patients twice and in 2 patients 3 times	The MSC group had a significantly higher Horovitz score of healthy lungs on discharge than the control group. Compared to controls, patients with MSC treatment showed a significantly lower Murray score of lung injury upon discharge than controls.
Yilmaz et al. [99] (*n* = 1)	Mesenchymal stem cells	MSC 1st application/day 1 3 × 10^6^/kg IV 2nd application/day 3 3 × 10^6^/kg IV 3rd application/day 6 3 × 10^6^/kg IV 4th application/day 9 2 × 10^6^/kg + 1 × 10^6^/kg intravenous + intrathecal	The application of MSCs has been found to have a healing effect on organs in this patient with severe COVID-19 infection.
Ping et al. [100] (*n* = 1)	Convalescent plasma and umbilical cord mesenchymal stem cells	6.5 × 10^7^ MSCs along with covalescent plasma	Intravenous infusion of CP and MSCs for the treatment of severe COVID-19 patients may have synergistic characteristics in inhibiting cytokine storm, promoting the repair of lung injury, and recovering pulmonary function
Lanzoni et al. [5] (*n* = 24)	Umbilical cord-mesenchymal stem cells	Subjects in the UC-MSC treatment group received two intravenous infusions of 100 ± 20 × 10^6^ UC-MSCs each, in 50 mL vehicle solution containing human serum albumin and heparin.	UC-MSC treatment was associated with a significant reduction in serious adverse events, mortality, and time to recovery, compared with controls. Treatment was associated with significantly improved patient survival (91% vs. 42%)
Tang et al. [101] (*n* = 2)	Mesenchymal stem cells	MSC infusion of 100 mL regardless of dose.	The fraction of inspired O2 (FiO2) gradually decreased while the oxygen saturation (SaO2) and partial pressure of oxygen (PO2) improved. Additionally, the patients' chest computed tomography showed that bilateral lung exudate lesions were adsorbed after MSC infusion.
Zhang et al. [102] (*n* = 1)	Human umbilical cord Wharton's jelly-derived mesenchymal stem cells	1 × 10^6^ cells per kilogram of weight of MSC	The percentage and counts of lymphocyte subsets (CD3+, CD4+, and CD8+ T cell) were increased, and the level of IL-6, TNF-*α*, and C-reactive protein is significantly decreased after hWJC treatment.
Feng et al. [103] (*n* = 16)	Umbilical cord mesenchymal stem cells	UC-MSCs of 1 × 10^8^ cells once. The patients would receive four rounds of transplantation in total, with one-day intervals in between.	Oxygenation index was improved, radiological presentations (ground glass opacity) were improved and the lymphocyte count and lymphocyte subsets (CD4+ T cells, CD8+ T cells, and NK cells) count showed recovery after transplantation.
Adas et al. [104] (*n* = 25)	Mesenchymal stem cells	The conventional treatment: piperacillin-tazobactam, favipiravir, dexamethasone, hydroxychloroquine, enoxaparine. Experimental group were administered 3∗10^6^ cell/kg MSC by intravenous infusion.	Conventional treatment with add-on MSC transplantation brought the cytokine storm under control and attenuate disease progression. MSC mediated growth and differentiation decreased the harm too, and accelerated the recovery of damaged organs resulting in reduced mortality, decreased ICU stay, and a promising safety profile.
Wei et al. [105] (*n* = 25)	Umbilical cord mesenchymal stem cells	1∗10^6^ cells/kg of MSCs along with conventional therapy vs. conventional therapy	The MSC-treated group demonstrated improved oxygenation index, reduction in the area of pulmonary inflammation, restoration of CT number in the inflamed area along with decreased IgM levels.
Meng et al. [74] (*n* = 18)	Human umbilical cord-derived mesenchymal stem cell	3 cycles of intravenous infusion of UC-MSCs (3 × 10^7^ cells per infusion) on days 0, 3, and 6 for treatment group along with standard COVID treatment regimens vs. standard treatment regimens only	Intravenous UC-MSCs infusion in patients with moderate and severe COVID-19 was safe and well tolerated
Kouroupis et al. [106] (*n* = 24)	Mesenchymal stem cells	UC-MSC iv infusion	UC-MSC recipients develop significantly increased levels of plasma sTNFR2 and significantly decreased levels of TNF*α* and TNF*β*, compared to controls indicating decrease of inflammation
Tao et al. [73] (*n* = 1)	Umbilical cord blood-derived mesenchymal stem cells	1.5 × 10^6^ USB-MSCs per kilogram of the patient's weight infused intravenously every 48 hours, with a total of five-time infusion.	USB-MSCs infusion, lymphocytes increased, and renal function improved, as well as pulmonary static compliance increased significantly and PaO2/FiO2 ratio maintained stable.
Primorac et al. [72] (*n* = 1)	Compassionate mesenchymal stem cell	10^6^ cells/kg of bone marrow-derived MSC on days 9, 12, and 16 days of hospitalization	MSC administration resulted in a reduction in leukocyte count, D-dimer levels, and CRP-levels, all of which are prognostic factors for COVID-19 severity.
Hashemian et al. [60] (*n* = 11)	Mesenchymal stem cells derived from perinatal tissues	3 intravenous infusions (200 × 10^6^ cells) every other day for a total of 600 × 10^6^ human umbilical cord MSCs (UC-MSCs; 6 cases) or placental MSCs (PL-MSCs; 5 cases).	Significant reductions in serum levels of tumor necrosis factor-alpha, IL-8, and C-reactive protein.

The article "Association between Mesenchymal Stem Cells and COVID-19 Therapy: Systematic Review and Current Trends" was published in 2022. Journal: Biomed Res Int.

**Table 2:** Summary of recruiting and not yet recruiting clinical trials involving use of mesenchymal stem cells in the treatment of COVID-19.

	Identifier	Study title	Cell therapy	Intervention (intravenous infusion)	Primary outcome
1	NCT04535856	Therapeutic Study to Evaluate the Safety and Efficacy of DW-MSC in COVID 19 Patients (*n* = 9)	Allogenic MSC low dose, high dose, and placebo	Drug; allogenic mesenchymal stem cell	Incidence of treatment-emergent adverse event in treatment group
2	NCT04313322	Treatment of COVID 19 Patients Using Wharton's Jelly-Mesenchymal Stem Cells (*n* = 5)	3 IV doses of WJ-MSCs consisting of 1∗10^6^/kg	Wharton's jelly-MSCs	Clinical outcomes followed by CT scan and RT-PCR
3	NCT04457609	Application of Umbilical Cord Mesenchymal Stem Cells as Adjuvant Therapy for Critically-Ill Patients (*n* = 40)	Umbilical cord-derived MSC/kg body weight in addition to standardised drugs.	Drug: oseltamivir Drug: azithromycin Biological: umbilical cord MSCs	Clinical improvement: presence of dyspnoea, sputum, fever, and ventilation status, blood pressure, heart rate, respiratory rate and oxygen saturation
4	NCT04525378	Mesenchymal Stromal Cell-based Therapy for COVID 19 associated Acute Respiratory Distress: a Pilot Clinical Study (*n* = 20)	MSC in low dose, intermediate dose, and doses	Mesenchymal stromal cell-based therapy	Intrahospital mortality within 28 days
5	NCT04269525	Clinical Research Regarding the Availability and Safety of UC-MSCs Treatment for Serious Pneumonia and Critical Pneumonia caused by 2019-nCOV Infection (*n* = 16)	UC-MSCs 3.3∗10^7^ cell number/50 mL/bag, on 1^st^, 3^rd^, 5^th^, and 7^th^ days after enrolment	Biological: umbilical cord-derived mesenchymal stem cells	Oxygenation index on day 14 after enrolment
6	NCT04397796	The Safety of Therapeutic Treatment with Immunomodulatory Mesenchymal Stem Cells in Adults with COVID 19 Infection Requiring Mechanical Ventilation (*n* = 45)	BM-Allo. MSC derived from bone marrow (CD73+, CD90+, CD105+, CD14-, CD34-, CD45-, and HLA-DR-)	Biological: BM-Allo. MSC	Incidence of adverse effects, mortality within 30 days, cause of death within 30 days, number of ventilation free days within 60 days of randomisation
7	NCT04903327	Treatment of COVID 19 Induced Acute Respiratory Distress: A Phase 2 Study of Intravenous Administration of Allogenic Adipose Derived Mesenchymal Stem Cells (*n* = 100)	COVI-MSC 2 vials on day 0, day 2, and day 4	Biological: COVI-MSC	All-cause mortality rate at day 28
8	NCT04467047	Safety and Feasibility of Allogenic Mesenchymal Stromal Cells in the Treatment of COVID 19 (*n* = 10)	1∗10^6^ MSCs/kg body weight mesenchymal stromal cell infusions	Biological: mesenchymal stromal cells infusion	Overall survival [time frame: 60 days]
9	NCT04452097	A Phase 1/2a Study of the Safety and Efficacy of BX-U001 for the Treatment of Severe COVID-19 Pneumonia with Moderate to Severe ARDS (*n* = 39)	Single infusion of hUC-MCS product at dose of 0.5 million cells/kg	Biological: human umbilical cord mesenchymal stem cells+ supportive care	Incidence of infusion-related adverse events [time frame-day 3] and incidence of any treatment emergent adverse events and treatment emergent serious adverse events [time frame: day 28]
10	NCT04444271	Prospective, Randomized Phase 2 Clinical Trial of MSCs for the Treatment of COVID-19 (*n* = 20)	Experimental: MSCs at dose 2∗10^6^/kg MSCs on day 1 and day 7 in addition to standard of care	Drug: mesenchymal stem cells	Overall survival [time frame-30 days postintervention]
11	NCT04390139	A Prospective Double-blind, Randomized, Parallel, Placebo controlled Pilot Clinical Trial for the Evaluation of the Efficacy and Safety of Two Doses of WJ-MSC in Patients with ARDS Secondary to Infection by COVID-19 (*n* = 30)	Experimental-Wharton-jelly MSCs on day 1 and day 3	Drug: XCEL-UMC-BETA	All-cause mortality at day 28
12	NCT04371393	Mesenchymal Stromal Cells for the Treatment of Moderate to Severe COVID-19 ARDS (*n* = 223)	Experimental-infusion of remestemcel-L 2∗10^6^ MSC/kg body weight plus standard of care	Biological: remestemcel-L Drug: placebo	Number of all-cause mortalities within 30 days of randomisation
13	NCT04339660	Clinical Research of Human MSCs in the Treatment of COVID-19 Pneumonia (*n* = 30)	Experimental: 1∗10^6^ cells/kg of weight of MSCs	Biological: UC-MSCs	The immune function-improvement and evaluative of pneumonia change
14	NCT04798716	MSC Exosomes for the Treatment of COVID-19 Positive Patients with ARDS and/or Novel Coronavirus Pneumonia (*n* = 55)	MSC-exosomes escalating dose every other day for a period of 5 days.	Drug: MSC-exosomes delivered IV every other day on escalating day	Treatment-related adverse events as assessed by CTCAE v4; for patients receiving ARDOXSO™, perinatal MSC-derived exosome therapy [time frame 90 days]
15	NCT04273646	Clinical Study of Human Umbilical Cord MSCs in the Treatment of Severe COVID 19 (*n* = 48)	Conventional treatment plus 4 times of UC-MSCs (0.5∗10^6^ UC-MSCs/kg body weight IV on day 1, 3, 5, and 7)	Biological: UC-MSCs Drug: placebo	Pneumonia severity index (time frame- 0 to 12 weeks after treatment) and oxygenation index (PaO2/FiO2)
16	NCT04537351	A Pilot, Open-label, Randomised Controlled Clinical Trial to Investigate Early Efficacy of CYP-001 in Adults Admitted to Intensive Care with Respiratory Failure (*n* = 24)	Experimental: CYP-001 IV infusion of 2 million Cymerus MSCs/kg body weight	Biological- CYP-001	Trend in trajectory of PaO2/FiO2 ratio [time frame- 7 days]
17	NCT04445220	A Multicentre, Randomised, Case controlled, Double-Blind, Ascending-dose study of Extracorporeal MSC in COVID-19 Subjects with Acute Kidney Injury Receiving Renal Replacement Therapy (*n* = 22)	Experimental: low dose and high dose SBI-101 device containing MSCs	Biological- SBI-101	Safety and tolerability as measured by incidence of IP-related serious adverse events [time frame- adverse events through day 180]
18	NCT04798066	HBPCOV01: Intermediate Size Patient Population Expanded Access Protocol to Evaluate the Safety and Efficacy of HB-adMSCs for the Treatment of Patients with Post COVID-19 Syndrome.	Autologous adipose-derived MSCs with a treatment duration of 14 weeks	Biological: HB-adMSCs	Treatment outcomes and adverse effects
19	NCT04456439	Intermediate size Expanded Access of Remesremcel-L, Human Mesenchymal Stromal Cells, for Multisystem Inflammatory Syndrome in Children Associated with Coronavirus Disease (COVID 19) (*n* = )	Remestecel-L – participants may receive upto 2 infusions of 2∗10^6^ L within a 5-day period Drug: hydrocortisone receiving and diphenhydramine receiving participants 30 minutes prior to the infusion of remestemcel-L	Biological: remestemcel-L Drug: hydrocortisone and diphenhydramine	Treatment outcomes and adverse effects
